# Development and Validation of a Prognostic Nomogram for Lung Adenocarcinoma: A Population-Based Study

**DOI:** 10.1155/2022/5698582

**Published:** 2022-12-10

**Authors:** Bin Xie, Xi Chen, Qi Deng, Ke Shi, Jian Xiao, Yong Zou, Baishuang Yang, Anqi Guan, Shasha Yang, Ziyu Dai, Huayan Xie, Shuya He, Qiong Chen

**Affiliations:** ^1^National Clinical Research Center for Geriatric Disorders, Xiangya Hospital, Central South University, Changsha 410008, China; ^2^Department of Geriatrics,Respiratory Medicine, Xiangya Hospital, Central South University, Changsha 410008, China; ^3^Department of Respiratory Medicine, Xiangya Hospital, Central South University, Changsha 410008, China; ^4^Department of Neurology, Xiangya Hospital, Central South University, Changsha 410008, China; ^5^Department of Geriatrics, Xiangya Hospital, Central South University, Changsha 410008, China; ^6^Department of Emergency Medicine, Xiangya Hospital, Central South University, Changsha 410008, China; ^7^Institute of Biochemistry and Molecular Biology, Hengyang Medical College, University of South China, Hengyang 421001, China

## Abstract

**Purpose:**

To establish an effective and accurate prognostic nomogram for lung adenocarcinoma (LUAD). *Patients and Methods*. 62,355 LUAD patients from 1975 to 2016 enrolled in the Surveillance, Epidemiology, and End Results (SEER) database were randomly and equally divided into the training cohort (*n* = 31,179) and the validation cohort (*n* = 31,176). Univariate and multivariate Cox regression analyses screened the predictive effects of each variable on survival. The concordance index (C-index), calibration curves, receiver operating characteristic (ROC) curve, and area under the ROC curve (AUC) were used to examine and validate the predictive accuracy of the nomogram. Kaplan–Meier curves were used to estimate overall survival (OS).

**Results:**

10 prognostic factors associated with OS were identified, including age, sex, race, marital status, American Joint Committee on Cancer (AJCC) TNM stage, tumor size, grade, and primary site. A nomogram was established based on these results. C-indexes of the nomogram model reached 0.777 (95% confidence interval (CI), 0.773 to 0.781) and 0.779 (95% CI, 0.775 to 0.783) in the training and validation cohorts, respectively. The calibration curves were well-fitted for both cohorts. The AUC for the 3- and 5-year OS presented great prognostic accuracy in the training cohort (AUC = 0.832 and 0.827, respectively) and validation cohort (AUC = 0.835 and 0.828, respectively). The Kaplan–Meier curves presented significant differences in OS among the groups.

**Conclusion:**

The nomogram allows accurate and comprehensive prognostic prediction for patients with LUAD.

## 1. Introduction

Lung cancer is the most common malignancy worldwide and is the leading cause of cancer-related death worldwide, accounting for 1.8 million deaths annually [1, 2]. Lung adenocarcinoma (LUAD) is the most common type of lung cancer, accounting for nearly 50% of non-small-cell lung cancers (NSCLC) [3, 4]. LUAD is characterized by a high degree of malignancy and poor prognosis [5]. In recent years, the incidence and mortality of LUAD have increased, despite the introduction of novel therapeutic approaches including immunotherapy or molecular targeted therapy [6, 7]. Recently, several prognostic factors for the survival of LUAD patients have been reported [8–10]. The studies mainly focused on LUAD-related genes and biomarkers, but these results lack the integration of some critical clinical information. Therefore, it is necessary to identify high-risk prognostic factors for predicting the individualized survival of patients with LUAD, and a nomogram is considered a good tool for predicting outcomes.

Nomograms, which can provide evidence-based, individualized, and highly accurate risk estimation, have been widely used for different types of cancer [11–13]. A nomogram is created by applying meaningful variables based on the results of regression analyses investigating potential prognostic factors, which contributed to better risk stratification and clinical decision-making [14–16]. The above makes the nomogram quite practical and easy to popularize.

The majority of previous nomograms in LUAD have focused on factors such as lesion size, lymph node metastasis, histological types, treatment factors, pathological stage, lymph node invasion, and age [17–19]. Nonetheless, there is a lack of comprehensive and accurate nomograms for predicting the survival of LUAD patients. The Surveillance, Epidemiology, and End Results (SEER) database is representative of the United States (US) population, with patient-level data abstracted from 18 geographically diverse populations including rural, urban, and regional populations [20]. It is widely used in cancer research [21, 22]. The SEER database contains rich information on LUAD patients; thus, it offers an excellent opportunity for LUAD study. Therefore, we used a cohort from the SEER database to develop a comprehensive, accurate, and effective nomogram for predicting the survival of LUAD patients.

## 2. Materials and Methods

### 2.1. Data Sources

Patients with LUAD were identified from the SEER database, a publicly available database, established in 1973. The database covers approximately 26% of the population of the US and includes 17 national population-based cancer registries [23]. Data from the SEER database includes demographic information as well as primary tumor site, tumor morphology, stage at diagnosis, the first course of cancer treatment, and follow-up information on the vital statistics of the patients with cancer. To include as much data as possible in the analysis, we retrieved database records from 1975 to 2016. All the patient information can be obtained from the supplementary section (supplementary 1. Date-AD and 2. Date-Code). (Available here).

### 2.2. Study Design

All included patients had data including definite LUAD diagnosis, age, sex, race, marital status, TNM staging, tumor size, grade, primary site, and overall survival (OS) information. LUAD was classified according to the International Classification of Diseases for Oncology, third edition (ICD-O-3), morphology codes: 8140, 8141, 8143, 8147, 8260, 8250–8257, 8323, 8480, 8481, 8550, 8570–8574, and 8576; and the site codes: C340–C343 and C348–C349. Patients with incomplete information listed above were excluded. The included patients were randomized into a training cohort (*n* = 31,179) and a validation cohort (*n* = 31,176) to develop and validate nomograms.

### 2.3. Statistical Analysis

All analyses were performed using R version 3.6.3 and R studio (https://www.r-project.org/). Cox regression analysis was used for univariate and multivariate analyses.

A nomogram was created based on the risk factors identified from the multivariate analysis using packages of “rms,” “foreign,” and “survival” in R studio. The performance of the model was measured using the concordance index (C-index), calibration curves, receiver operating characteristic (ROC) curve, and the area under the ROC curve (AUC). The larger the C-index, the more accurate the prognostic prediction [24]. We use the “predict” function in the “survival” R package to calculate the risk score of the samples in the training cohorts. Based on the median risk score, the samples were then divided into a high-risk group and a low-risk group. Survival curves were constructed using the Kaplan–Meier method and compared using the log-rank test. During the internal validation of the nomogram, the C-index, calibration curves, and ROC curves were derived from the regression analysis using the same R package described above. A *P* value < 0.05 was considered statistically significant.

## 3. Results

### 3.1. Clinical Characteristics of Patients

A total of 67,146 patients with LUAD were identified from the SEER database. Of these, 62,355 patients who satisfied the inclusion criteria were enrolled and randomly divided into the training (*n* = 31,179) and validation (*n* = 31,176) cohorts. The methods used for data collection and analysis are summarized in Figure 1. The clinical characteristics of patients are listed in Table 1.

### 3.2. Independent Prognostic Factors in the Training Cohort

The results of the univariate and multivariate analyses are presented in Table 2. The multivariate analyses demonstrated that age, sex, race, marital status, AJCC-N, AJCC-M, tumor size, grade, and the primary tumor site were independent risk factors for OS.

### 3.3. Prognostic Nomogram for OS

The nomogram was constructed using all significant independent factors derived from the regression analysis above and the AJCC-T (an important aspect of AJCC-TMN staging) for OS in the training cohort (Figure 2). The C-index of this model for OS prediction was 0.777 (95% confidence interval (CI), 0.773 to 0.781). Furthermore, the calibration plot for the probability of survival at 3 or 5 years presented good agreement between nomogram prediction and actual observation (Figures 3(a) and 3(b)). AUC for the 3- and 5-year OS was 0.832 and 0.827 in the training cohort (Figures 4(a) and 4(b)), respectively, showing good accuracy of the nomogram.

### 3.4. Validation of the Nomogram

In the validation cohort, the C-index of this model for OS prediction was 0.779 (95% CI, 0.775 to 0.783), slightly higher than that of the training cohort. The calibration curves also presented good agreement between prediction and observation for the 3- and 5-year survival probabilities (Figures 5(a) and 5(b)). The ROC curves showed good accuracy of the nomogram for predicting 3- or 5-year OS, as shown in Figures 6(a) and 6(b) (AUC = 0.835 and 0.828, respectively).

### 3.5. Survival and Prognostic Factors for OS

The Kaplan–Meier analysis was conducted to identify vital prognostic factors that could be useful to predict the outcome. The effects of vital factors for predicting OS across all patients with LUAD are shown in Figure 7. We found survival rates were significantly higher in the low-risk group than in the high-risk group (Figure 7(a)). As shown in Figure 7(b), patients aged 60–69 years had the best survival, but patients over 80 years had the worst survival. Survival for the other age groups was between patients aged 60–69 years and patients over 80 years, in order of worsening survival, 50–59, <50, and 70–79 (*P* < 0.0001). Male patients presented better survival than female patients (*P* < 0.0001) (Figure 7(c)). Further analysis showed that other races were associated with better outcomes compared with white and black races (*P* < 0.0001) (Figure 7(d)). Married patients (including married and domestic partners) showed better survival than single patients (including single, widowed, divorced, and separated), as shown in Figure 7(e) (*P* < 0.0001). Better survival was observed in LUAD stage T1 than in other stages (Figure 7(f)) (*P* < 0.0001). Different from the T stage, patients in the N0 stage exhibited better survival than in the N1, N2, or N3 stages (Figure 7(g)) (*P* < 0.0001). The survival probability in the M0 stage was higher than in the M1 stage (including M1a and M1b) (Figure 7(h)) (*P* < 0.0001). As illustrated in Figure 7(i), the smaller the tumor size, the better the survival generally. However, the not otherwise specified (NOS) group presented the worst survival probability (*P* < 0.0001). In the plot association between grade level and survival, grade I had better survival than other grades (Figure 7(j)) (*P* < 0.0001). However, patients with grade IV tumors achieved better survival than grade III patients. In Figure 7(k), patients with the primary site at the middle lobe showed better survival than those with primary sites at the lower lobe, upper lobe, overlapping lesion of the lung, lung NOS, or the mainstem bronchus (*P* < 0.0001).

## 4. Discussion

LAUD is a highly heterogeneous tumor in terms of pathology, biology, and clinical behavior, which leads to significant challenges to therapy and prognostic prediction [25, 26]. In the past, several different approaches have been attempted to predict the prognosis of LAUD patients, for example, using features from pathology images, molecule biomarkers based on bioinformatics analysis and laboratory data, and clinical staging [27–29]. Here, our research focused on the combination of pathology, bioinformatics, and clinical characteristics of LAUD patients and provided a more accurate assessment of the prognosis of LAUD patients. We considered a nomogram to be an appropriate choice.

In our study, we evaluated the prognostic factors in the SEER database using Cox regression analysis (Tables 1 and 2). The SEER database provides a public population-based database, which means less inconsistency than that of institutions [30, 31]. In our study, age, sex, race, marital status, TNM stages, tumor size, grade, and primary site were considered and identified as predictors of OS in patients with LAUD (Tables 1 and 2). With increasing T stages, hazard ratio (HR) values increased, although *P* values were not significant in the multivariate Cox regression analyses. We think the few patients in the T0 stage (*n* = 19) in the training cohort may be attributed to the result (Table 1). Nonetheless, T staging still plays a crucial role in predicting the survival of lung cancer patients [32, 33]. Thus, we took the AJCC-T stage into account for the construction of the nomogram to avoid any inappropriate exclusion of this variable. In addition, we used the AJCC 8th Edition for lung cancer to precisely classify the lesion sizes of LUAD patients and to define the relationship between tumor size and prognosis. The nomogram was then constructed based on the training cohorts to predict the 3- and 5-year OS of LAUD patients (Figure 1). The nomogram we established was more targeted for LUAD patients than the nomogram established for non-small-cell lung cancer (NSCLC) patients [34]. The C-index of the nomogram was 0.777 (95% CI, 0.773 to 0.781) in the training cohorts, indicating a good concordance between prediction and actual OS. Furthermore, we found a good concordance in the calibration curves (Figures 2(a) and 2(b)) as well as for the ROC curves (Figures 3(a) and 3(b), AUC = 0.832 and 0.827, respectively) for 3- and 5-year OS. All these results illustrated that the nomogram model achieved good predictive accuracy. We considered the relatively high predictive accuracy of the nomogram from three aspects. First, we choose an appropriate method, univariable and multivariable Cox regression analyses, to analyze the relationship between predictive factors and prognosis. Second, the predictive factors we chose and identified are more closely associated with each LAUD patient. Most of these variables had been reported in previous studies as risk factors for NSCLC survival [35–41]. Thus, our nomogram integrated these closely related factors for all LAUD patients. Other factors, such as chronic obstructive pulmonary disease (COPD), cigarette smoking, and surgery, are not required for all LAUD patients [33]. So, we did not include those risk factors in the analysis. Third, to some extent, the large number of patients included in the analysis contributed to the accuracy of the model.

The C-index, calibration curves, ROC curves, and AUC values were also used to validate the predictive accuracy of the nomogram in the validation cohorts. The C-index was 0.779 (95% CI, 0.775 to 0.783) in the validation cohort, which was higher than the training cohort. The calibration lines overlapped more closely to the standard lines than the training cohort (Figures 4(a) and 4(b)). The AUC values under the ROC curves for the 3- and 5-year OS showed better concordance in the validation than in the training cohort (Figures 5(a) and 5(b), AUC = 0.835 and 0.828, respectively). Hence, in the current study, the C-indexes, calibration plots, ROC curves, and AUC values showed optimal agreement between prediction and actual observation, guaranteeing the repeatability and reliability of the constructed nomogram. Overall, the nomogram was able to predict the prognosis of LUAD patients effectively and precisely.

However, the primary limitation of our research is the lack of external validation. Some studies have examined the generalizability of their constructed nomograms via external validation [42]. But our model is based on a large set of globally representative data, which enhances its generalizability. Our use of random sampling and effective internal verification ensured the accuracy of the prediction. At the same time, it is relatively difficult to collect enough LUAD patients for external validation in a short time. Larger multicenter studies will be needed in the future due to the lack of external validation in our study.

Furthermore, we investigated the impact of prognostic factors on patient survival. The cutoff value of the risk score determined by the Cox regression analyses was used to stratify patients into two groups. Patients with a low-risk score (≤0.798) presented better survival, similar to previous studies on LUAD and NSCLC [42, 43]. In addition, according to the Kaplan–Meier analysis, age, sex, race, marital status, TNM stage, tumor size, grade, and primary tumor site were associated with survival.

The age stratification in our study was more detailed than in other studies, which is more conducive to analyzing the effect of different ages on patient survival. In our study, we concluded that age was closely correlated with LUAD survival. Older age predicted lower OS, which is consistent with other studies [44]. Furthermore, we demonstrated that female patients showed better survival, which is consistent with previous studies [45]. However, different results have been reported on whether age and sex have an impact on the survival of patients with LUAD. In the study by Pitz et al., sex but not age was an independent factor affecting prognosis, and women with LUAD showed better survival than men [46]. In contrast, Jubelirer et al. concluded that age, not sex, was the significant prognostic factor for LUAD [47]. Surprisingly, Zhao et al. concluded that neither age nor sex was a significant prognostic factor for LUAD patients [48]. We consider that these disagreements arose from an analysis of different databases or differences in study objectives.

The impact of race on the survival of patients with lung cancer has been reported previously. Several lines of evidence have suggested that races other than white and black had the best survival [23, 49]. The same trend was observed in our study. However, it is controversial whether the white or black race can be associated with lower survival. Data from several studies demonstrated there was no significant difference in survival between white and black patients with lung cancer [23, 50]. Nonetheless, our study and other studies have reported that black patients with lung cancer experienced worse survival rate than white patients [49, 51]. Some evidence indicates that white patients may have a worse survival rate [52]. The great differences in smoking prevalence and hospital choices between black and white patients may partly explain these differences [53, 54].

It has been reported that marital status was a protective factor for survival among patients with lung cancer [55, 56]. The married patients in our study included married couples and those living with domestic partners, and singles were defined as single, widowed, divorced, and separated patients, which was a more detailed definition than previous studies [56, 57]. We highlighted the potentially significant social impact of marital status on the survival of LUAD patients. In the present study, a higher survival rate was shown in married patients. Similar results have been observed in other cancers, such as pancreatic and liver cancer [58, 59].

The TNM staging system is widely accepted as a tool to predict the prognosis of patients with cancer and provide therapy guidelines to doctors. Here, we did not include patients with stage Tx or Nx when assessing the impact of factors on prognosis to guarantee more accuracy and avoid potential errors caused by overdetailed classifications. Although the Kaplan–Meier curves showed that the higher T stage shortened the survival of the patients, patients at the T0 stage did not present the best survival in our study. We speculated that this is because of the lack of sufficient patients at the T0 stage. Patients at the N0 stage had better survival than those at higher N stages as shown in previous studies [60]. That means that lymph node metastasis exerted a negative impact on the survival of LUAD patients. The same tendency was also observed for patients at the M stage, that distant metastasis of LUAD reduces the survival rate. The same conclusion can be obtained from other studies [61]. Thus, higher TNM stages indicate poorer survival of LUAD patients.

We further confirmed the effect of tumor size on prognosis based on the 8th edition of the AJCC. Compared with the 7th edition, the latest staging criteria place greater emphasis on the importance of tumor size for a patient's prognosis [62, 63]. Hence, using the most recent criteria, one can effectively analyze the effect of tumor size on prognosis. In the present study, smaller tumor size was associated with a better prognosis, while the NOS group presented the worst. A previous study also established that the tumor size in lung cancer was negatively correlated with survival [23]. However, a majority of studies have not considered the NOS group [51]. We attributed this phenomenon to the complex workup and uncertain classification of the NOS group. Taken together, our specific classification in tumor size made it suitable to predict the prognosis of LUAD patients.

To date, several studies have indicated that the differentiation of the tumor was associated with survival in patients with lung cancer [64, 65]. The general rule emerging from these studies was that the poorer the differentiation of the tumor, the shorter the survival of the patients with lung cancer. Our results validated most of these findings. However, to our surprise, tumors with grade IV differentiation showed even better survival than grade III. We attributed this difference to the limited number of patients in grade IV included in our study (*n* = 288). More patients in grade IV should be included in the future study.

Previous studies have explored the relationship between the primary site of NSCLC and prognosis [66]. However, conclusions from clinical studies remain controversial. Wang et al. reported that patients with lung cancer in the lower lobe had worse survival than tumors in the upper lobes [67]. Li et al. demonstrated that patients with NSCLC located in the main bronchus experienced worse outcomes than at other locations [68]. However, some studies have indicated that the primary site could not contribute to predicting the survival of NSCLC at stages I/II [69]. In the current study, we found that patients with lower and upper lobe tumors showed poorer survival than middle lobe tumors, and mainstem bronchus tumors showed the worst prognosis. Different from the grouping used in previous studies, we added the NOS group to provide additional guidelines for LUAD patients. The survival time of the lung NOS group fell between the mainstem bronchus and overlapping lesions of the other lung groups. Overall, this evidence suggests that the tumor primary site has a significant impact on prognosis and should be considered in prognosis assessment.

## 5. Conclusion

In conclusion, we established and validated a novel nomogram for predicting the survival of LUAD patients. Younger age, female sex, race other than white and black, married status, lower risk score, lower TNM staging, smaller tumor size, and high differentiation grade of the tumor were associated with good survival. Using this model, clinicians may evaluate the survival of LUAD individuals more precisely. In the future, the underlying mechanisms leading to these results should be studied to improve our understanding of LUAD.

## Figures and Tables

**Figure 1:** Data analysis workflow.

**Figure 2:** Lung adenocarcinoma survival nomogram. A nomogram-predicted survival risk based on age, sex, and other factors in patients with lung adenocarcinoma. A patient's value is located on each variable axis, and the score corresponds to the number on the top line.

**Figure 3:** Calibration curves for training cohort. The calibration curves for predicting the overall survival of patient at (a) 3 and (b) 5 years in the training cohort. Nomogram-predicted probability of overall survival and actual survival proportion is plotted on the *x*-axis and *y*-axis, respectively.

**Figure 4:** Receiver operating characteristic curves for training cohort. Receiver operating characteristic (ROC) curves for (a) 3 and (b) 5 years in the training cohort.

**Figure 5:** Calibration curves for validation cohort. The calibration curves for predicting the overall survival of patient at (a) 3 and (b) 5 years in the validation cohort. Nomogram-predicted probability of overall survival and actual survival proportion is plotted on the *x*-axis and *y*-axis, respectively.

**Figure 6:** Receiver operating characteristic curves for validation cohort. Receiver operating characteristic (ROC) curves for (a) 3 and (b) 5 years in the validation cohort.

**Figure 7:** Kaplan–Meier survival curves of the training cohort. Kaplan–Meier survival curves for the training cohort on the basis of the nomogram. (a) Risk level; (b) age; (c) gender; (d) race; (e) marital status; (f) AJCC-T stage; (g) AJCC-N stage; (h) AJCC-M stage; (i) tumor size; (j) grade; (k) primary site.

**Table 1:** Clinical characteristics of patients with lung adenocarcinoma.

Variables	Total (*n* = 62355)	Training cohort (*n* = 31179)	Validation cohort (*n* = 31176)
Age (years), *n* (%)			
<50	2469 (3.96)	1246 (4.00)	1223 (3.92)
50–59	10101 (16.20)	5109 (16.39)	4992 (16.01)
60–69	19589 (31.42)	9762 (31.31)	9827 (31.52)
70–79	20425 (32.76)	10200 (32.71)	10225 (32.80)
≥80	9771 (15.67)	4862 (15.59)	4909 (15.75)
Sex, *n* (%)			
Female	33618 (53.91)	16768 (53.78)	16850 (54.05)
Male	28737 (46.09)	14411 (46.22)	14326 (45.95)
Race, *n* (%)			
Black	6773 (10.86)	3372 (10.81)	3401 (10.91)
White	50222 (80.54)	25170 (80.73)	25052 (80.36)
Others	5360 (8.60)	2637 (8.46)	2723 (8.73)
Marital status, *n* (%)			
Married	35027 (56.17)	17527 (56.21)	17500 (56.13)
Single	27328 (43.83)	13652 (43.79)	13676 (43.87)
AJCC_T, *n* (%)			
T0	43 (0.07)	19 (0.06)	24 (0.08)
T1	21609 (34.65)	10722 (34.39)	10887 (34.92)
T2	19632 (31.48)	9892 (31.73)	9740 (31.24)
T3	10844 (17.39)	5392 (17.29)	5452 (17.49)
T4	10227 (16.40)	5154 (16.53)	5073 (16.27)
AJCC_N, *n* (%)			
N0	36208 (58.07)	18112 (58.09)	18096 (58.04)
N1	5687 (9.12)	2847 (9.13)	2840 (9.11)
N2	15450 (24.78)	7743 (24.83)	7707 (24.72)
N3	5010 (8.03)	2477 (7.94)	2533 (8.12)
AJCC_M, *n* (%)			
M0	42862 (68.74)	21459 (68.83)	21403 (68.65)
M1	19493 (31.26)	9720 (31.17)	9773 (31.35)
Tumor size (cm), *n* (%)			
≤3	32231 (51.69)	15990 (51.28)	16241 (52.09)
3–5	14814 (23.76)	7483 (24.00)	7331 (23.51)
5–7	6715 (10.77)	3362 (10.78)	3353 (10.76)
≥7	5070 (8.13)	2564 (8.22)	2506 (8.04)
NOS	3525 (5.65)	1780 (5.71)	1745 (5.60)
Grade, *n* (%)			
I	11626 (18.64)	5783 (18.55)	5843 (18.74)
II	24877 (39.90)	12427 (39.86)	12450 (39.93)
III	25328 (40.62)	12681 (40.67)	12647 (40.57)
IV	524 (0.84)	288 (0.92)	236 (0.76)
Primary site, *n* (%)			
Mainstem bronchus	940 (1.51)	482 (1.55)	458 (1.47)
Upper lobe	35977 (57.70)	17968 (57.63)	18009 (57.77)
Middle lobe	3150 (5.05)	1589 (5.10)	1561 (5.01)
Lower lobe	18737 (30.05)	9336 (29.94)	9401 (30.15)
Overlapping lesion of lung	623 (1.00)	309 (0.99)	314 (1.01)
Lung NOS	2928 (4.70)	1495 (4.79)	1433 (4.60)

AJCC_T, American Joint Committee on Cancer_Tumor; AJCC_N, American Joint Committee on Cancer_Node; AJCC_M, American Joint Committee on Cancer_Metastasis; NOS, not otherwise specified.

**Table 2:** Univariate and multivariate Cox regression analyses in the training cohort.

Variables	Univariate			Multivariate		
	HR	95% CI	*P* value	HR	95% CI	*P* value
Age (years)						
<50	Ref			Ref		
50–59	1.021	0.938–1.110	0.637	1.245	1.144–1.355	<0.001
60–69	0.947	0.874–1.026	0.184	1.386	1.278–1.503	<0.001
70–79	1.083	1.000–1.174	0.049	1.817	1.670–1.970	<0.001
≥80	1.512	1.391–1.643	<0.001	2.529	2.325–2.751	<0.001
Sex						
Female	Ref			Ref		
Male	1.454	1.411–1.498	<0.001	1.401	1.358–1.445	<0.001
Race						
Black	Ref			Ref		
Others	0.716	0.667–0.768	<0.001	0.736	0.686–0.790	<0.001
White	0.848	0.810–0.889	<0.001	0.989	0.944–1.038	0.661
Marital status						
Married	Ref			Ref		
Single	1.190	1.155–1.226	<0.001	1.250	1.211–1.290	<0.001
AJCC_T						
T0	Ref			Ref		
T1	0.444	0.246–0.803	0.007	1.080	0.596–1.960	0.799
T2	0.868	0.480–1.568	0.639	1.193	0.657–2.165	0.562
T3	1.357	0.751–2.453	0.312	1.328	0.732–2.410	0.351
T4	1.971	1.091–3.562	0.025	1.401	0.772–2.541	0.267
AJCC_N						
N0	Ref			Ref		
N1	1.889	1.793–1.990	<0.001	1.401	1.328–1.478	<0.001
N2	3.353	3.239–3.471	<0.001	1.701	1.636–1.770	<0.001
N3	4.479	4.265–4.704	<0.001	1.743	1.651–1.841	<0.001
AJCC_M						
M0	Ref			Ref		
M1	4.949	4.798–5.105	<0.001	3.023	2.912–3.139	<0.001
Tumor size (cm)						
≤3	Ref			Ref		
3–5	2.003	1.929–2.080	<0.001	1.244	1.185–1.306	<0.001
5–7	2.962	2.828–3.103	<0.001	1.396	1.320–1.477	<0.001
≥7	3.555	3.381–3.737	<0.001	1.591	1.497–1.692	<0.001
NOS	5.692	5.384–6.017	<0.001	1.878	1.758–2.007	<0.001
Grade						
I	Ref			Ref		
II	1.478	1.407–1.553	<0.001	1.237	1.177–1.301	<0.001
III	2.922	2.787–3.064	<0.001	1.710	1.626–1.798	<0.001
IV	2.725	2.353–3.155	<0.001	1.613	1.392–1.870	<0.001
Primary site						
Mainstem bronchus	Ref			Ref		
Upper lobe	0.327	0.297–0.361	<0.001	0.750	0.680–0.828	<0.001
Middle lobe	0.311	0.276–0.349	<0.001	0.731	0.649–0.823	<0.001
Lower lobe	0.324	0.293–0.358	<0.001	0.775	0.701–0.857	<0.001
Overlapping lesion of lung	0.484	0.410–0.571	<0.001	0.878	0.744–1.037	0.126
Lung NOS	0.757	0.678–0.847	<0.001	0.845	0.755–0.946	0.003

AJCC_T, American Joint Committee on Cancer_Tumor; AJCC_N, American Joint Committee on Cancer_Node; AJCC_M, American Joint Committee on Cancer_Metastasis; NOS, not otherwise specified; HR, hazard ratio; CI, confidence intervals; Ref, reference.

## Data Availability

The data used to support the findings of this study are from publicly available datasets and are available at https://seer.cancer.gov/data/.

## Supplementary Materials

Supplementary Materials The first Excel table named “1. Date-AD” in the supplementary materials section contains all the patient information sorted out, such as age and gender. The second Excel table named “2. Date_Code” is the code used to convert the data downloaded from the public data into a useable format.
